The article "Asiaticoside, a trisaccaride triterpene induces biochemical and molecular variations in brain of mice with parkinsonism" was retracted in 2024. Reasons: duplicated images; overlap with earlier publications; unreliable results or conclusions; concerns about the images.

# Asiaticoside, a trisaccaride triterpene induces biochemical and molecular variations in brain of mice with parkinsonism

**DOI:** 10.1186/2047-9158-2-23

**Published:** 2013-11-21

**Authors:** Uvarajan Sampath, Vanisree Arambakkam Janardhanam

**Affiliations:** 1 Department of Biochemistry, Indo-American College, Cheyyar, Tamilnadu, India; 2 Department of Biochemistry, University of Madras, Guindy Campus, Chennai, Tamilnadu, India

## Abstract

**Background:**

Parkinson’s disease characterized by oxidative stress and mitochondrial damage in the pars compacta of substantia nigra remains a challenge to manage with an added disadvantage of side effects of L-levo dopa, the standard drug used for therapy. Thus, an alternative approach of utilizing natural components would be beneficial in the management of the disease. The present study was aimed to investigate the potential role of asiaticoside (As), a trisaccaride triterpene against1 – methyl 4 – phenyl 1,2,3,6 tetrahydropyridine (MPTP)-induced neurotoxicity in experimental mice.

**Methods:**

Mice were divided into 4 groups: Group I received vehicle saline, group II was treated with 20 mg/kg of body weight of MPTP (2 doses with 2 h intervals), group III received MPTP along with 50 mg/kg body weight of As for the 21 consecutive days starting from the day of MPTP intoxication. Group IV received 50 mg/kg body weight of asiaticoside for the same period serving as drug control. Animals were sacrificed at the end of experimental period and the striatum and midbrain samples were analyzed for enzyme assays, transmission electron microscopic (TEM) analysis. Immunofluorescent assay was performed to study the expression of GFAP to detect astrocyte, which are activated due to neuronal damage. Imunohistochemical studies were carried out to quantify the expression of Bax and Bcl2, the molecular signatures that would provide clues of the extent of neurodegeneration.

**Results:**

The activities of enzymes were increased on As administration when compared with those of group II animals. Expressions of Bax and Bcl2 along with GFAP did show significant variations (p < 0.05) on MPTP treatment when compared to control animals and the changes were found to be reversed significantly (p < 0.05) after treatment with asiaticoside. TEM analysis also showed attenuated degenerative architecture on As administration. The mice which received As alone (drug control IV) did not show significant variation from that of the control mice.

**Conclusion:**

The observations suggest that asiaticoside may be efficacious in protecting neurons from the oxidative damage caused by the insult of MPTP.

## Introduction

Parkinson’s disease (PD) is one of the major neurodegenerative disorders. The etiology of this disease is likely due to the combinations of environmental and genetic factors. Symptomatic hallmarks of PD are tremor, bradykinesia, rigidity and postural instability. PD is characterized by massive degeneration of dopaminergic neurons in the substantia nigra pars compacta (SNpc), leading to a severe loss of striatal dopaminergic fibers and to a massive reduction of dopamine levels in the striatum [1]. The neurons project their axons to the striatum and utilize dopamine as their neurotransmitter [2] and a profound reduction in striatal dopamine represents the primary neurochemical alteration in PD. The proapoptotic protein Bax is highly expressed in the SNpc and if reduced would attenuate SNpc developmental neuronal apoptosis [3]. PD involving such pathology is the second largest intimidating health hazard next to Alzeimer’s disease and is currently being managed by drugs such as Levodopa which only aid in symptomatic relief.

Among various therapeutic strategies, the intake of antioxidants through dietary or pharmacological could reduce the oxidative stress induced by various degenerating neurotoxins. Literature survey showed evidences of protective action of *Centella asiatica* (CA) against MPTP induced parkinsonism in rats [4]. Traditionally the leaves and stems of CA are used for various medicinal purposes. CA was found to protect against monosodium glutamate induced neurodegeneration owing to its potential antioxidant property [5]. It was found to be effective in preventing the cognitive deficits, as well as the oxidative stress caused by intracerebroventricular administration of streptozotocin, indicating that CA can act as a free radical scavenger [6]. Further CA was found to increase brain GABA levels in rat models [7]. Asiaticoside (As) and Asiatic acid (Aa) are the two major active principles that have been isolated from CA. Asiaticoside derivatives were found to inhibit or reduce H_2_O_2_ induced cell death and lower intracellular free radical concentration, protecting aginst the effects of beta-amyloid neurotoxicity [8].

With such baseline informations on PD pathology and on asiaticoside, whose mechanisms of neuroprotective action need to be explored, the current study has been designed with the hypothesis that Asiaticoside, the active principle of CA could have an impact on parkinosnic features in mice.

Thus, the study aims at the exploration of the effect of asiaticoside against MPTP –induced neurotoxicity in mice, by evaluating the critical features such as activities of ATPases, expressions of Bax and Bcl2 and astrocyte activation which are established by the researchers as hallmarks of neurodegeneration.

## Materials and methods

### Reagents

MPTP – HCl and asiaticoside were purchased from sigma – Aldrich Bangalore. All the Chemicals used for the study were of analytical grade. Karnovsky’s fixative, Araldite CY212 (10 ml), DDSA (dodecenylsuccinic anhydride) DMP (dimethyl aminomethyl phenol) (0.4 ml), plasticizer, Uranyl acetate and Lead citrate were used for electron microscopic analysis.

### Animals

Swiss albino mice (BALB/c) (8 – 14 weeks old) weighing about the 25 – 30 g of weight were used for the study. Animals were purchased from Tamilnadu Veterinary and Animal science University (TANUVAS), Madhavaram, Chennai, India and were housed under standard conditions of temperature (26 ± 1°C) and illumination (12 h light/dark cycles), water and standard rodent food *ad libitum*. The protocol was approved by the Institutional Animal Ethics Committee of the University of Madras. (IAEC NO; 01-078-09).

### Experimental protocol

The mice were injected intraperitoneally (i.p.) with two administrations of MPTP (20 mg/kg) at 2-h intervals, the total dose per mice being 40 mg/kg. A total of 24 animals were divided into four groups: group I was treated with 2 ml of 0.9% NaCl and served as control; group II received MPTP – HCl (i.p.) at the dosage of 20 mg/kg of two doses at 2 h interval and served as PD model; group III treated with MPTP-HCl (i.p) along with 50 mg/kg body weight of asiaticoside (orally) for 21 consecutive days; group IV received 50 mg/kg body weight of asiaticoside (orally) served as drug control. Following the toxicity assessment of both acute and sub chronic [9] studies, the dosage of 50 mg/kg body weight of asiaticoside was fixed for the current study. Animals were sacrificed at the end of the experimental period.

### Brain tissue collection

The mice were sacrificed by cervical decapitation in the morning to avoid diurnal variations of the endogenous amines, enzymes and other antioxidant molecules. Striatal and mid brain portions were separated and weighed. The brain tissues were excised and examined under microscope ensuring the sections**.** The sections were homogenized (approx. 10% weight/volume) in 0.32 M sucrose and centrifuged at 1000 \ g for 10 min to remove cell debris and nuclei. The supernatant was collected and recentrifuged at 1000 \ g for another 10 min. The resulting supernatant was layered over 1.2 m sucrose, and centrifuged at 34,000 \ g for 50 min at 4°C. The fraction collected between the 0.32 m and 1.2 m sucrose layer was diluted at 1:1.5 with ice-cold bi-distilled water, further layered on 0.8 m sucrose, and again centrifuged at 34,000 \ g for 30 min. The pellet thus obtained was washed, repelleted at 20,000 \ g for 20 min, and ruptured with ice-cold 5 mm imidazole-HCl buffer, pH 7.4 and kept in ice for 60 min with occasional vortex at high speed every 5 min and used for enzyme assay [10].

### Estimation of ATPases

The activity of Na+/K + ATPases, Ca2+ ATPase and Mg2+ ATPase were evaluated [11-13] in the brain samples. Normalization in ATPase detection was done by total protein estimation. The level of total protein was estimated with bovine serum albumin (BSA) as the standard [14].

### Statistics

All the grouped data were expressed as mean ± SD. Difference in means was studied by means of ANOVA followed by Dunnet’s post hoc test. Results were considered significant at p < 0.05.

### Immunohistochemistry studies

The tissue sections were deparaffinized in xylene I & xylene II at 60°C for 20 min each and hydrated through a graded series of alcohol, the slides were incubated in a citrate buffer (pH 6.0) for three cycles of 5 min each in a microwave oven for antigen retrieval. The sections were then allowed to cool to room temperature and then rinsed with TBS, and treated with 0.3% H_2_O_2_ in methanol for 10 min to block endogenous peroxidase activity. Non-specific binding was blocked with 3% BSA at room temperature for 1 h. The sections were then incubated with diluted primary antibody Bax (1:1000), Bcl-2 (1:1000) from spring Bioscience USA. The slides were washed with TBS and then incubated with anti – rabbit/anti mouse HRP – labeled secondary antibody (Genei, Bangalore, India) at a dilution (1:500) for 1 h in room temperature. The peroxidase activity was visualized by treating the slides with 3, 3′ – diaminobenzidine tetrahydrochloride (SRL, Mumbai, India); the slides were counterstained with Meyer’s hematoxylin. Negative controls were incubated with TBS instead of primary antibodies. The relative intensive scoring was done by arbitrary units (i.e. number of positive cells per 40× field).

### Immunofluorescence study for GFAP

Immunofluorescence was performed on the striatal and mid brain portion of brain tissues. Tissue samples were fixed in 10% buffered formalin and embedded in paraffin wax. Sections were cut at 5 μm in thickness and deparaffinized in two changes of xylene at 600C for 20 min each and hydrated through a graded series of alcohol, the slides were incubated in a citrate buffer (pH 6.0) for three cycles of 5 min each in a microwave oven for antigen retrieval. These sections were then allowed to cool to room temperature and then rinsed with TBS and treated with 0.3% H_2_O_2_ in methanol for 10 min to block endogenous peroxidase activity. Non specific binding was blocked with 3% BSA at room temperature for 1 h. The sections were then incubated with following diluted primary antibodies GFAP (1:100) at 40°C overnight. The slides were washed with TBS and then incubated with anti-mouse FITC (fluorescence isothiocyanate) –labeled secondary antibody (Genei, Bangalore, India) at a dilution 1:500 for 30 min in room temperature. Then they were washed thrice with TBS and mounted in glycerol: PBS mix (1:9). Then slides were viewed under fluorescence microscope using wavelength of 590 nm.

### Transmission electron microscopy (TEM)

The samples were fixed in Karnovsky’s fixative for 6 – 8 h at 4°C. These were post fixed in 1% Osmium tetraoxide in 0.1 M phosphate buffer for 2 h at 4°C, dehydrated in ascending grades of acetone, infiltrated and embedded in araldite CY212 and polymerized at 60°C for 72 h. Thin (60 – 70 nm) sections were cut with an ultra – microtome. The sections were mounted on copper grids and stained with urany1 acetate and lead citrate and observed under a transmission electron microscope.

## Results

Table 1 illustrates the activity of membrane bound enzymes namely Na^+^K^+^, Mg2^+^, Ca2^+^ ATPases which were significantly reduced (p < 0.05) in the striatum and midbrain of MPTP induced mice (Group II) when compared to group I. The activities of ATPases were reported after normalization of level of total protein. Upon the administration of As (Group III), the activities of these enzymes were increased when compared with those of group II animals. The mice which received As (drug control IV) did not show significant variation from that of the control mice (Table 1).

**Table 1:** **Effect of As on the activities of Na**^**+**^**K**^**+ **^**ATPase, Mg**^**2+ **^**ATPase, Ca**^**2+ **^**ATPase in the striatal and midbrain tissue of control and experimental mice**

	**Striatal tissue**				**Midbrain**			
**Particulars**	**Group I** **(Control)**	**Group II** **(MPTP induced)**	**Group III** **(MPTP induced + AS Treated)**	**Group IV** **(AS Control)**	**Group I** **(Control)**	**Group II** **(MPTP induced)**	**Group III** **(MPTP induced + AS Treated)**	**Group IV** **(AS Control)**
Na^+^ K ^+^ ATPase	0.33 ± 0.01	0.25 ± 0.03^a*^	0.33 ± 0.04^b*^	0.34 ± 0.06^NS^	0.34 ± 0.13	0.23 ± 0.03^a*^	0.34 ± 0.02^b*^	0.34 ± 0.02^NS^
Mg^2+^ ATPase	0.44 ± 0.03	0.32 ± 0.02^a*^	0.35 ± 0.03^b*^	0.44 ± 0.04^NS^	0.44 ± 0.03	0.35 ± 0.06^a*^	0.43 ± 0.02^b*^	0.45 ± 0.02^NS^
Ca^2+^ ATPase	0.54 ± 0.06	0.34 ± 0.04^a*^	0.35 ± 0.03^b*^	0.44 ± 0.08^NS^	0.54 ± 0.08	0.33 ± 0.01^a*^	0.46 ± 0.01^b*^	0.56 ± 0.02^NS^

Na^+^ K ^+^, Mg^2+^, Ca^2+^ ATPase = μmoles of Pi liberated/min/mg protein. Each value expressed as mean ± S.D for six mice (n = 6) in each group. Statistically significance at *p < 0.05; a group I *vs* group II, b group II vs group III and (NS) non-significant group IV vs group I.

Bax is a protein of Bcl -2 gene family which promotes apoptosis. Figures 1 and 2 represent the immunohistochemical staining pattern of Bax in the striatum and midbrain respectively of control and experimental groups. Similarly, Figures 3 and 4 represent the expression of bcl2 in straitum as well as midbrain respectively. The corresponding scoring of the expression pattern were represented as arbitrary units in Figure 5 (Bax) and 6 (Bcl 2). MPTP induced mice (Group II) showed a significant reduction (p < 0.05) in the number of positively cells of Bcl2 (Figures 3 and 4), when compared with those of control (Group I), while As treatment significantly (p < 0.05) increased the number of positive cells in Bcl2 when compared with that of group I. In contrast to the above observation, an increased number of Bax positive cells was found in MPTP induced mice (Group II) [as compared to group I] and the same was reversed upon the treatment of As. Figure 5 and 6 shows the Densitometric pattern of the expression of Bax and Bcl 2 in striatum and midbrain respectively.

**Figure 1:** **Immunohistochemical expression pattern of Bax in striatum. A**: Control (group1); **B**: MPTP induced (group II); **C**: MPTP induced + As treated (group III); **D**: Drug Control (group IV).

**Figure 2:** **Immunohistochemical expression pattern of Bax in mid brain. A**: Control (group 1); **B**: MPTP induced (group II); **C**: MPTP induced + As treated (group III); **D**: Drug Control (group IV).

**Figure 3:** **Immunohistochemical expression pattern of Bcl-2 in striatum. A**: Control (group 1); **B**: MPTP induced (group II); **C**: MPTP induced + As treated (group III); **D**: Drug Control (group IV).

**Figure 4:** **Immunohistochemical expression pattern of Bcl-2 in mid brain. A**: Control (group 1); **B**: MPTP induced (group II); **C**: MPTP induced + As treated (group III); **D**: Drug Control (group IV).

**Figure 5:** **Each bar represented the mean ± S.D of 6 mice (n = 6).** * represents statically significance at P < 0.05. Comparasion were made as (a) group I vs group II, (b) group II vs group III, (c) group I vs group III, (#) non significant group I vs group IV (scale bar 50 μm) **A**: Densitometric pattern of the expression of BAX in the striatum. **B**: Densitometric pattern of the expression of BAX in the midbrain.

**Figure 6:** **Each bar represented the mean ± S.D of 6 mice.** * represents statistically significant at P < 0.05. Comparasion were made as (a) group I vs group II, (b) group II Vs group III, (c) group I vs group III, (#) non significant group I vs group IV (scale bar 50 μm) **A**: Densitometric pattern of the expression of Bcl 2 in striatum. **B**: Densitometric pattern of the expression of Bcl 2 in midbrain.

### Immunofluorescence of GFAP

Figures 7 and 8 represent the immunofluorescence pattern of GFAP in striatum and mid brian respectively of the experimental mice. Prominent expression of GFAP was encountered on MPTP intoxication owing to reactive astrogliosis following the insult by MPP^+^. The sections from As treated mice did show a comparative reduction in the immunofluorescence of the protein under investigation suggesting the lesser impact of the insult. Figure 9 shows the Densitometric pattern of the expression of GFAP in striatum and midbrain.

**Figure 7:** **Depict the immunofluorescent pattern of GFAP positive cells in striatum and midbrain respectively, exhibiting markedly increased, ramified form with many fine processes in MPTP treated mice.** GFAP immunoreactivity was mild in the striatum and midbrain of control (Group I) and AS treated mice (Group III). Immunoflurosence expression of GFAP in striatal tissue. **A**: Control (group 1); **B**: MPTP induced (group II); **C**: MPTP induced + As treated (group III); **D**: Drug Control (group IV).

**Figure 8:** **Depict the immunofluorescent pattern of GFAP positive cells in striatum and midbrain respectively, exhibiting markedly increased, ramified form with many fine processes in MPTP treated mice.** GFAP immunoreactivity was mild in the striatum and midbrain of control (Group I) and AS treated mice (Group III). Immunoflurosence expression of GFAP in mid brian tissue. **A**: Control (group 1); **B**: MPTP induced (group II); **C**: MPTP induced + As treated (group III); **D**: Drug Control (group IV).

**Figure 9:** **Each bar represented the mean ± S.D of 6 mice (n = 6).** * represents statistical significant at P < 0.05. Comparasion were made as (a) group I vs group II, (b) group II Vs group III, (c) group I vs group III, (#) non significant group I vs group IV (scale bar 50 μm) **A**: Densitometric pattern of the expression of GFAP in striatum. **B**: Densitometric pattern of the expression of GFAP in midbrain.

### Transmission electron microscopy

Figures 10 and 11 depict the ultra structural architecture of striatal tissue and midbrain viewed under transmission electron microscope. Control mice (Group I) showed normal nuclei and cytoplasm similar to that of drug control (Group IV). In MPTP induced mice, striatum and midbrain (Group II) showed enlarged axon and neuron fibers displaying abnormal dense filamentous material, autophagic structure and irregular multi vesicular bodies (arrow) chromatin condensation was also encountered. MPTP induced As treated mice (Group III) showed lesser intensity of the above mentioned changes.

**Figure 10:** **Transmission electron microscopic appearance of striatum. A**: Transmission electron microscopic appearance of striatum Control (group1); **B1**: low resolution of MPTP induced (group II); **B2**: high resolution of MPTP induced (group II); **C**: MPTP induced + As treated (group III); **D**: Drug Control (group IV).

**Figure 11:** **Transmission electron microscopic appearance of midbrain. A**: Transmission electron microscopic appearance of midbrain Control (group 1); **B1**: low resolution of MPTP induced (group II); **B2**: high resolution of MPTP induced (group II); **C**: MPTP induced + As treated (group III); **D**: Drug Control (group IV).

## Discussion

MPTP is oxidized by monoamine oxidase B (MAO-B) to a 1-methyl-4-phenyl-pyridinium (MPP^+^). MPP^+^ is looked upon as the toxic substrate, which inhibits complex I activity in mitochondria [15]. An additional toxic mode of action involves the dopamine transporter, which carries MPP^+^ in dopaminergic neurons [16].

Na^+^K^+^ –ATPase is the enzyme responsible for the active transport of sodium and potassium ions in the nervous system, maintaining and re-establishing, after each depolarization, the electrochemical gradient necessary for neuronal excitability and regulation of neuronal cell volume. This enzyme is present in high concentrations in brain cellular membranes, consuming about 40 – 50% of the ATP generated in this tissue [17]. The enzyme is known to be affected by the redox state of the cell and reduced antioxidants or antioxidant enzymes activities are related to reduced Na^+^ K^+^ - ATPase activity [18-20]. By this, ROS are believed to be involved in tissue damage, resulting in a wide variety of insults [21-23]. Inhibition of Na^+^K^+^ - ATPase activity is found in various neuropathological conditions, including cerebral ischemia [24] and neurodegenerative disorders [25-27]. MPTP treated mice shown decreased ATPase activity the same was significantly reversed upon by As treatment.

Bcl-2, an anti–apoptotic member of the Bcl–2 family can bind to Bax to form Bcl–2: Bax heterodimers attenuate the pro–apoptotic effect of Bax [28]. Bcl–2 and Bax are involved in the regulation of caspase–3 mediated apoptosis [29]. Bcl–2 can inhibit apoptosis by binding to the pro – apoptotic Bax, Bcl–xs, and Bad proteins; it is believed that the Bcl–2/ Bax ratio is a determining factor for the cell’s fate [30,31]. MPTP is known to decrease the expression of Bcl–2 and increased expression of Bax in the striatum [32] thereby tilting the balance towards apoptosis. MPTP administration could induce a cell apoptosis in PD model [33] via its active MPP^+^ from an impairing mitochondrial function. The subsequent energy failure with ATP depletion increases formation of free radicals [34] and cytochrome C release [35,36]. It is reported that the primary cultured neurons which over–express Bcl–2 could be resistant to the toxicity of MPTP [37]. The study exhibited a comparative increase in the expression of BCl-2 and the decrease in that of Bax (Group III) suggesting that As could minimize the effects of MPTP by an yet -to -identify mechanism.

Astrocytes secrete various neurotoxic substances and express an enhanced level of glial fibrillary acidic protein (GFAP), which is considered a marker protein for astrogliosis [38]. GFAP- positive astrocytes were evident in the striatum and midbrain portions after the MPTP treatment (Group II, B) as the latter could cause astroglial activation. These results provide valuable information for the pathogenesis of acute stage of Parkinson’s disease [39,40]. Astrocytes react to various neurodegenerative insults rapidly, leading to vigorous astrogliosis [41,42]. This intensified astrocytic activation was not observed in As treatment (Figures 7 and 8) suggesting the minimal insult by MPTP in As treated mice and hence minimal reactive astrocytes.

Transmission electron microscopic view of the sections of striatum and midbrain of As treated mice depicts minimal abnormal variations such as irregular multi vesicular bodies and dense filamentous material when compared to group II where these changes were more prominent as seen in Figures 10 and 11. This observation suggests the neuro-shielding potential of As against MPTP intoxication in the mice.

The study thus highlights the potential of As to minimize the Bax which is required for death of neurons that activates downstream effectors of cell death such as caspases [43], with a concomitant increase in the anti-apototic Bcl2 [44] by an yet to prove mechanism leading to protection of cells. By this and also due to the improved activities of ATPases, As might influence the translocation of transmitters, nutrients, ions, and cellular components between different cellular compartments that could be beneficial for neuronal integrity as evidenced from the results. Further, the astroglial activation by MPTP was only less pronounced by As. Thus, asiaticoside, a triterpenoid of Centella asiatica is found to have significant neuroprotective mechanism against MPTP – induced neurotoxicity and thus could be considered as a potential candidate for further evaluation against Parkinsonism.

## Abbreviations

PD: Parkinson disease; As: Asiaticoside; MPTP: 1 – methyl 4 – phenyl 1,2,3,6 tetra hydro pyridine; GFAP: Glial fibrillary acidic protein; BCL 2: B cell lymphoma 2; GABA: Gama amino butyric acid.

## Competing interests

The authors declare that they have no competing interests.

## Authors’ contributions

All the works except GFAP have been done by US. GFAP has done by VAJ. Both authors read and approved the final manuscript.
